The article "Automatic Diagnosis of Mild Cognitive Impairment Based on Spectral, Functional Connectivity, and Nonlinear EEG-Based Features" was published in 2022. Journal: Comput Math Methods Med.

# Automatic Diagnosis of Mild Cognitive Impairment Based on Spectral, Functional Connectivity, and Nonlinear EEG-Based Features

**DOI:** 10.1155/2022/2014001

**Published:** 2022-08-11

**Authors:** Reza Akbari Movahed, Mohammadreza Rezaeian

**Affiliations:** Department of Biomedical Engineering, Hamedan University of Technology, Hamedan, Iran

## Abstract

Accurate and early diagnosis of mild cognitive impairment (MCI) is necessary to prevent the progress of Alzheimer's and other kinds of dementia. Unfortunately, the symptoms of MCI are complicated and may often be misinterpreted as those associated with the normal ageing process. To address this issue, many studies have proposed application of machine learning techniques for early MCI diagnosis based on electroencephalography (EEG). In this study, a machine learning framework for MCI diagnosis is proposed in this study, which extracts spectral, functional connectivity, and nonlinear features from EEG signals. The sequential backward feature selection (SBFS) algorithm is used to select the best subset of features. Several classification models and different combinations of feature sets are measured to identify the best ones for the proposed framework. A dataset of 16 and 18 EEG data of normal and MCI subjects is used to validate the proposed system. Metrics including accuracy (AC), sensitivity (SE), specificity (SP), F1-score (F1), and false discovery rate (FDR) are evaluated using 10-fold crossvalidation. An average AC of 99.4%, SE of 98.8%, SP of 100%, F1 of 99.4%, and FDR of 0% have been provided by the best performance of the proposed framework using the linear support vector machine (LSVM) classifier and the combination of all feature sets. The acquired results confirm that the proposed framework provides an accurate and robust performance for recognizing MCI cases and outperforms previous approaches. Based on the obtained results, it is possible to be developed in order to use as a computer-aided diagnosis (CAD) tool for clinical purposes.

## 1. Introduction

Dementia is the most prominent neurological disorder among the elderly, resulting in deterioration of cognitive abilities such as memory, thinking, behavior, and limitation in performance of daily activities [1]. While dementia mostly affects people over the age of sixty, some individuals are afflicted with this condition at a younger age. It was estimated that 44.4 million people around the world suffer from some forms of dementia [2, 3]. Alzheimer's disease (AD) is the most common type of dementia, comprising about 60% to 80% of dementia cases [4]. AD causes severe memory loss, cognitive impairment, and behavioral changes. In the United States, it is the third most costly illness and the sixth most common cause of mortality [4]. Unfortunately, there is no effective treatment for AD and anti-AD medications merely serve to alleviate the symptoms of the disease. Hence, diagnosis of AD at an early stage is essential for controlling the progress of the disease. Mild cognitive impairment (MCI) is the intermediate stage between the normal cognitive deficit due to aging and AD or other forms of dementia, and it is frequently considered the early stage of AD. It is estimated that about 15% to 20% of dementia cases lead to AD [5]. According to some experts, diagnosis of MCI is more critical than AD, because it is more optimum to the management of the disease at the MCI stage. A more accurate method for diagnosis of MCI is therefore crucial to the control of disease progress. Nonetheless, the symptoms of MCI are often indistinguishable from those associated with growing older. Diagnosis of MCI was done integrating multiple experiments including psychological tests such as mini-mental state examinations (MMSE), blood tests, spinal fluid analysis, neurological examination, and magnetic resonance imaging (MRI). However, these traditional methods are laborious, time-consuming, and error prone. Therefore, many MCI cases may not be diagnosed accurately and in a timely fashion. Hence, novel and automated methods for early and accurate MCI diagnosis are in high demand. Electroencephalography (EEG) is an efficient modality which records the bioelectrical activity of brain neurons corresponding to various states from the scalp surface area. EEG signals can depict the functioning of the brain with great temporal resolution and are noninvasive, inexpensive, and portable for recording. As a result, it might be employed as a biological biomarker for MCI and other types of dementia that is objective and trustworthy. The manual interpretation of these signals is tough and challenging due to their nonstationary and nonlinearity nature. Many researchers are urged to employ machine learning techniques for automated EEG signal analysis in light of the advancements in computer science and artificial intelligence. For instance, numerous studies have been conducted to automatically detect different neurological disorders such depression [6–8], epilepsy [9–11], seizure [12–15], Parkinson's disease [16, 17], and schizophrenia [18].

The article "Automatic Diagnosis of Mild Cognitive Impairment Based on Spectral, Functional Connectivity, and Nonlinear EEG-Based Features" was published in 2022. Journal: Comput Math Methods Med.

EEG-based machine learning frameworks for diagnosing AD, MCI, and other forms of dementia have been reported in a number of research [19–28]. An automatic MCI diagnosis method, for instance, was presented by Kashefpoor et al. [19] and is based on the extraction of spectral characteristics of EEG signals. This method involved extracting 19 spectral features from 19-channel EEG data based on the delta, theta, alpha1, alpha2, gamma, beta1, and beta2 frequency subbands. The best discriminative features were then chosen using a correlation-based feature selection algorithm. The classification test was carried out using the neuro-fuzzy (NF) and k-nearest neighbor (KNN) classifiers, and an accuracy of 88.89% was reported in their study as the best classification result. Using spectrum and complexity analysis, McBride et al. proposed an EEG-based classification framework that distinguishes between AD, MCI, and healthy individuals [20]. The complexity analysis comprises computational activity, mobility, complexity, sample entropy, and Lempel-Ziv complexity parameters. The spectral analysis involves extracting features from the delta, theta, alpha1, alpha2, gamma, beta1, and beta2 frequency subbands. In this work, an average accuracy of 79.2% was obtained for MCI classification using the support vector machine (SVM) classifier. In a different study, Kashefpoor et al. used 19-channel EEG signals along with supervised dictionary learning techniques like label consistent K-SVD (LC-KSVD) and correlation-based label consistent K-SVD (CLC-KSVD) to diagnose MCI [21]. On two separate dictionary learning classifiers, they applied a time series signal as well as a vector of retrieved spectral features. By casting a vote between the predictions of the time series signal and spectral characteristic vector, the final forecast for each sample was determined. The CLC-KSVD approach yielded an accuracy of 88.9%, which is the highest achieved accuracy in this investigation. A single-channel EEG-based technique for MCI diagnosis using speech-evoked brain responses was presented by Khatun et al. [22]. Using time and spectral domain analysis to extract 590 characteristics from the recorded sounds, the top 25 were chosen using the random forest (RF) method. They used logistic regression (LR) and support vector machine (SVM) classification models for the classification task, and the best classification result that they found was an accuracy of 87.9%. Based on the spectral-temporal analysis, Yin et al. proposed an integrated MCI diagnosis approach in [23]. This method uses spectral-temporal analysis to extract a collection of features and then uses a developed wrapper algorithm called the three-dimensional (3-D) evaluation algorithm to derive an ideal feature subset. The SVM classifier in this investigation had the best accuracy rate, which was 96.94%. Power spectral density (PSD), skewness, kurtosis, spectral skewness, spectral kurtosis, spectral crest factor, spectral entropy (SE), and fractal dimension (FD) properties were used by Sharma et al. to construct an automatic EEG-based MCI detection technique [24]. The study's dataset was gathered under four different conditions: open eyes, closed eyes, the finger tapping test (FTT), and a continuous performance test (CPT). The SVM classifier achieved the best classification accuracy of this method, which was 96.94%. Fast Fourier transform (FFT) and wavelet transform (WT) feature extraction techniques were used by Durongbhan et al. in [25] to offer an automatic AD detection methodology based on EEG recordings. The presented findings show that this method used the KNN classifier to achieve an accuracy of 99%. Using the piecewise aggregate approximation (PAA) compression approach and feature extraction techniques like permutation entropy (PE) and autoregressive (AR), Siuly et al. created a system for automatically identifying MCI patients [26]. The classification models utilized in this investigation were the extreme learning machine (ELM), SVM, and KNN. According to the presented data, the ELM classifier had the best classification performance thanks to its accuracy of 98.78%. Using the interhemispheric coherence features and the properties of EEG subbands, Oltu et al. proposed another EEG-based paradigm for the classification of MCI, AD, and healthy people [27]. For feature extraction, this method used the discrete wavelet transform (DWT), PSD, and interhemispheric coherence; for classification, it used bagged trees. The best outcome of this study was 96.5%. Another strategy for differentiating between AD and healthy participants using EEG data was put out by Safi and Safi [28]. This method involved applying the DWT, PSD, and empirical mode decomposition (EMD) algorithms to the signals and then extracting certain features from the outputs of the aforementioned algorithms, including variance, kurtosis, skewness, Shannon entropy, sure entropy, and Hjorth parameters. This study compared SVM, KNN, and regularized linear discriminant analysis (RLDA) and found that KNN had the greatest classification performance with an accuracy of 97.64%.

The article "Automatic Diagnosis of Mild Cognitive Impairment Based on Spectral, Functional Connectivity, and Nonlinear EEG-Based Features" was published in 2022. Journal: Comput Math Methods Med.

A viable and accurate method for clinical usage has not yet been provided, despite the fact that numerous studies on automated EEG-based MCI diagnosis have been carried out. In other words, achieving an optimal/robust performance with high accuracy, which might be used for clinical applications, is the main problem of autonomous EEG-based MCI diagnosis. So, based on EEG signals, we present a precise machine learning-based methodology for MCI detection. To do this, EEG data are processed to extract three key feature sets, including spectral, functional connectivity, and nonlinear properties. The sequential backward feature selection (SBFS) technique is used to choose the optimal feature combination. To select the optimal categorization model for the suggested methodology, various models are evaluated. Additionally, each feature set and its combinations with other feature sets are investigated in the suggested technique to determine which combination is optimal. Additionally, the most important functional connectivity aspects as well as EEG signal strength disparities in common EEG frequency subbands between MCI and HC patients were also looked into.

## 2. Materials and Methodology

### 2.1. Dataset

A public dataset consists of EEG recorded signals from MCI patients and healthy control participants, provided by Kashefpoor et al. [21], was utilized in this investigation. It contains 18 EEG data from MCI patients and 16 EEG data from healthy participants. This dataset's participants were all older than 55. At Noor Hospital in Isfahan, Iran, these participants were identified and chosen. This hospital also performed neuropsychological examinations, EEG recordings, and other experimental procedures. The individuals' diagnoses and the experimental design for data gathering were authorized by the ethics committee of the vice chancellor's office at the Isfahan University of Medical Sciences for Research and Technology in Isfahan, Iran. Based on Peterson's criteria, participants' MCI diagnoses were made. 19 EEG electrodes were put in accordance with the 10-20 International System to record EEG data from each subject while they were all resting and their eyes were closed (Fp1, Fp2, F7, F3, Fz, F4, F8, T3, C3, Cz, C4, T4, T5, P3, Pz, P4, T6, O1, and O2). For 30 minutes, these signals were collected. Additionally, the electrode-skin impedance was less than 5 k*Ω*, and the sampling rate was set to 256 Hz.

### 2.2. Proposed Methodology

The proposed methodology for MCI diagnosis based on EEG data is summarized in Figure 1. Preprocessing, feature extraction, feature selection, classification, and validation make up the proposed methodology. The EEG signals underwent preprocessing to remove noise and artifacts. In this step, each signal was sliced into one-minute segments after suppressing noise and artifacts. Then, using EEG segments, the spectral, functional connectivity, and nonlinear feature sets were retrieved. Following that, 10-fold crossvalidation was used to randomly divide the samples into the training and testing sets. To choose the most effective discriminative features, the training set was used during the feature selection process. The feature selection algorithm in this work was the SBFS approach. The training set was then used to train the classifier after the nonselected features had been eliminated from the testing and training sets. The trained classification model was then used to classify each case of the testing set for validating the suggested methodology.

The article "Automatic Diagnosis of Mild Cognitive Impairment Based on Spectral, Functional Connectivity, and Nonlinear EEG-Based Features" was published in 2022. Journal: Comput Math Methods Med.

#### 2.2.1. Preprocessing

Eye movements, eye blinks, electromyogram (EMG), electrocardiograms, electrode channel drift, and power line interference are just a few of the noise and aberrations that can contaminate EEG signals and prohibit a pure portrayal of brain function in the data. In order to prevent further inaccurate analysis, it is crucial to remove noise and artifacts from the EEG signal. Using the EEGLAB toolbox in MATLAB, a preprocessing approach was conducted to all recorded EEG signals in this investigation [29]. A band-pass filter with a low cutoff frequency of 0.5 Hz and a high cutoff frequency of 32 Hz was used to filter the signals in the first step. Due to the components of the aforementioned artifacts being focused outside the frequency band between 0.5 Hz and 32 Hz, it reduces the effects of EMG and power line interference. The independent components of the signals were then extracted using the independent component analysis (ICA) methodology, and using a voting classification method, each component was classified into artifact and nonartifact classes. The ICLabel [30] and MARA [31] automatic plugins, along with manual inspection, projected a label for each component in this voting classification approach, and the final predicted label was the one that obtained more than half of the votes. The signals were then rebuilt after the expected artifact components had been removed. The remaining noisy intervals were then taken out of the reconstructed signals using a visual analysis. Finally, to increase the amount of samples, the preprocessed EEG signals were sliced into one-minute segments using a nonoverlapping sliding window. It should be noted that the labels on the EEG data segments matched those on the EEG signal's original label.

#### 2.2.2. Feature Extraction

By converting each raw sample's values into a select few useful features, feature extraction in machine learning is aimed at representing each sample with the qualities that are task relevant. The spectral, functional connectivity, and nonlinear feature sets are extracted from the EEG segments using the suggested methods. The explanation of each extracted feature set is as follows:

1. *Spectral features*: the spectral properties of the EEG signals are intended to depict the characteristics of the frequency subbands of the EEG at various scalp locations. Due to their relation to brain's function, these characteristics may serve as diagnostic criteria for neurological illnesses. In this study, the spectral feature set was created by extracting the band power of each EEG segment's interhemispheric asymmetry and theta (4 to 8 Hz), alpha (8 to 13 Hz), and beta (13 to 32 Hz) frequency subbands. To determine the band power of frequency subbands, the PSD of EEG segments was calculated using the Welch periodogram [32]. The Hamming window with a 50% overlap between the windows was used in the Welch periodogram. It is important to note that each channel of the EEG segments was used to extract the band powers of the aforementioned frequency subbands. The definition of interhemispheric asymmetry, which measures disparities in the band power of the frequency subbands in the left and right hemispheres, is as follows:

(1) $$\begin{array}{c} IA=\log\left(P_{RH}\right)-\log\left(P_{LH}\right), \end{array}$$

where *IA*, *P*_*RH*_, and *P*_*LH*_ stand for the interhemispheric asymmetry, the band power in the right hemisphere, and the band power in the left hemisphere, respectively. The interhemispheric asymmetry for the channel pairings Fp2-Fp1, F4-F3, F8-F7, C4-C3, T4-T3, P4-P3, T6-T5, and O2-O1 was computed in this work for the delta, theta, alpha, and beta frequency subbands

(2) *Functional connectivity features*: numerous research has looked at brain connection in recent years to understand how information is processed, sent to, received by, or shared between various brain regions during various cognitive tasks and mental states. A branch of neuroscience known as functional connectivity seeks to quantify the statistical relationships between the dynamics of concurrently recorded signals [33] in order to gauge brain connectivity. Coherence, mutual information, and synchronization likelihood are only a few examples of functional connectivity metrics used to assess brain connectivity. Here, a collection of characteristics based on the statistical correlations between EEG channels in various scalp areas was extracted using the synchronization likelihood method [34]. In general, synchronization likelihood analyzes the nonlinear and linear dependencies between two signals, which may be complex and significantly different in the two signals, to estimate the synchronization between them. The possibility of synchronization between two signals is represented numerically by a value between zero and one. More synchronization between two signals is indicated by a greater value for this metric. First, a time-delay embedding method that is specified as follows [34] was used to create a state-space representation of an M-channel EEG signal:

(2) $$\begin{array}{c} X_{k,i}=\left[x_{k,i},x_{k,i+l},\cdots ,x_{k,i+\left(m-1\right)l}\right], \end{array}$$

where *kε*{1, 2, ⋯, *M*}, *iε*{1, 2, ⋯, *N*}, *m*, *l* are the channel number, the index of each discrete sample, embedding dimension, and lag parameters, respectively. Next, (*P*_*k*,*i*_^*ε*^) is defined as follows to state that *X*_*k*,*i*_ and *X*_*k*,*j*_ vectors are closer than a distance of *ε* [34].

(3) $$\begin{array}{c} P_{k,i}^{\varepsilon }=\frac{1}{2\left(\omega_{1}-\omega_{2}\right)}\overset{N}{\underset{j=1}{\sum }}\phi \left(\varepsilon -\left|X_{k,i}-X_{k,j}\right|\right),\;\omega_{1}<\left|i-j\right|<\omega_{2}, \end{array}$$

where *ϕ*, |.|, *ω*_1_, and *ω*_2_ stand for Heaviside step function, Euclidean distance, dimension of the Theiler correction window, and dimension of the sharpening window, respectively. Each of the Theiler and sharpening windows establish a window around the discrete sample *i* to modify autocorrelation consequences and sharpen the time resolution of the synchronization measure. Now, *ε*_*k*,*i*_ is determined for each *k* and each *i* for which *P*_*k*,*i*_^*ε*_*k*,*i*_^ = *p*_ref_, where *p*_ref_ ≪ 1. In the next step, the number of channels where the *X*_*k*,*i*_ and *X*_*k*,*j*_ will be closer together than *ε*_*k*,*i*_(*H*_*i*,*j*_) is determined for each sample pair (*i*, *j*) and within the considered window (*ω*_1_ < |*i* − *j*| < *ω*_2_) as follows [34]:

(4) $$\begin{array}{c} H_{i,j}=\overset{M}{\underset{k=1}{\sum }}\phi \left(\varepsilon_{k,i}-\left|X_{k,i}-X_{k,j}\right|\right). \end{array}$$

*H*_*i*,*j*_ indicates how many of the embedded time series signals resemble each other, and it varies between 0 and *M*. Now, the synchronization likelihood for each channel (*k*) and each discrete sample pair (*i*, *j*), (*S*_*k*,*i*,*j*_) is defined in (5) [34].

(5) $$\begin{array}{c} S_{k,i,j}=\left\{\begin{array}{cc} \frac{H_{i,j}-1}{M-1}, & \text{if }\left|X_{k,i}-X_{k,j}\right|<\varepsilon_{k,i},\\ 0, & \text{if }\left|X_{k,i}-X_{k,j}\right|>\varepsilon_{k,i}. \end{array}\right. \end{array}$$

To obtain the rate of synchronization between channel *k* at sample *i* and all other *M* − 1 channels (*S*_*k*,*i*_), an averaging over all *j* of *S*_*k*,*i*,*j*_ is performed as follows [34]:

(6) $$\begin{array}{c} S_{k,i}=\frac{1}{2\left(\omega_{1}-\omega_{2}\right)}\overset{N}{\underset{j=1}{\sum }}S_{k,i,j},\;\omega_{1}<\left|i-j\right|<\omega_{2}. \end{array}$$

*S*_*k*,*i*_ ranges between *p*_ref_ and 1. *S*_*k*,*i*_ = 1 indicates the maximum synchronization of all *M* channels, and *S*_*k*,*i*_ = *p*_ref_ corresponds with the case where all *M* channels have minimum synchronization. Finally, the average of *S*_*k*,*i*_ over all *i* is computed and expressed as synchronization likelihood between *k* channels. In this work, *p*_ref_, *l*, *m*, *ω*_1_, and *ω*_2_ were set to 0.01, 10, 10, 100, and 410, respectively, and the synchronization likelihood between the same channels was not calculated. It is worth mentioning that these paraments were chosen using trial and error experiments to obtain the most reasonable connectivity image

(3) *Nonlinear features*: EEG signals by their very nature have complicated behavior and nonlinear dynamic properties. In light of this, nonlinear analysis techniques may be superior than conventional linear analysis techniques for describing EEG signals. In this study, certain nonlinear features, including detrended fluctuation analysis, Higuchi fractal properties, correlation dimension, Lyapunov exponent, C0-complexity, Kolmogorov entropy, Shannon entropy, and approximate entropy, were computed from each channel of the EEG segments. The features are each further detailed in the paragraphs as follows
  - *Detrended fluctuation analysis*: it is an algorithm for estimating the statistical self-affinity of a time series [35]. Consider a finite signal, *x*(*t*) of length *N*. First, a summation version of *x*(*t*) is obtained as follows:

(7) $$\begin{array}{c} X\left(k\right)=\overset{k}{\underset{i=1}{\sum }}\left(x\left(i\right)-\overset{¯}{x}\right), \end{array}$$

where $\overset{¯}{x}$ is the mean value of *x*(*t*). Next, *X*(*k*) is segmented into the *n* windows with equal lengths and a least-square line is calculated by minimizing the squared errors within each window. *Y*_*n*_(*k*) denotes the resulting least-square line fitting. Then, the root-mean-square deviation from the trend, the fluctuation, is computed as follows:

(8) $$\begin{array}{c} F\left(n\right)=\sqrt{\frac{1}{N}\overset{N}{\underset{k=1}{\sum }}\left(X\left(k\right)-Y_{n}\left(k\right)\right)}, \end{array}$$

where *F*(*n*) is the fluctuation. Finally, the computing of (8) is replicated for windows with different sizes to form a logarithmic scale of *F*(*n*) against *n*. It can be denoted by *F*(*n*) = *n*^*α*^, in which *α* represents the self-affinity of the signal. In other words, *α* is the extracted feature by detrended fluctuation analysis

(b) *Higuchi fractal properties*: Higuchi proposed an algorithm to calculate the fractal dimension of a signal in 1988 [36]. Given a signal with *N* samples (*x*(*t*)), *T* new signals are generated using the following equation:

(9) $$\begin{array}{c} X_{\tau }^{T}=\left\{x\left(\tau \right),x\left(\tau +T\right),\cdots ,x\left(\tau +\left[\frac{N-\tau }{T}\right]\right)\right\}, \end{array}$$

where *τ* = 1, 2, ⋯, *T* and [*r*] denotes the integer part of *r*. Let *L*_*τ*_(*T*) represent the length of each signal which is defined as follows:

(10) $$\begin{array}{c} L_{\tau }\left(T\right)=\frac{1}{T}\frac{\sum_{i=1}^{\left[\left(N-\tau \right)/T\right]}\left|x\left(\tau -iT\right)-x\left(\tau \left(i-1\right)T\right)\right|\times \left(N-1\right)}{\left[\left(N-\tau \right)/T\right]}. \end{array}$$

Also, *L*(*T*) is defined to obtain the mean length for each signal as follows:

(11) $$\begin{array}{c} L\left(T\right)=\overset{T}{\underset{\tau =1}{\sum }}L_{\tau }\left(T\right). \end{array}$$

Finally, (11) is computed for all *T* values ranging from *T*_min_ to *T*_max_ and the slope of the linear fitting of ln*L*(*T*) versus ln1/*T* is considered as the Higuchi fractal dimension of *x*(*t*). In this study, the *T*_min_ and *T*_max_ were set to 1 and 30 values, respectively. These parameters were selected such that the Higuchi fractal characteristic could be extracted from the study's data

(c) *Correlation dimension*: it is another approach for calculating the fractal dimension by measuring the occupied space by a set of random points. In 1983, Grassberger and Procacia presented a method for computing correlation dimension, which is the most common method for estimating correlation dimension [37]. Firstly, it constructs an *m*-dimensional vector using time delay (*τ*) and embedding dimension (*m*), which can be denoted as follows:

(12) $$\begin{array}{c} X\left(i\right)=\left[x\left(i\right),x\left(i+\tau \right),\cdots ,x\left(i+\left(m-1\right)\tau \right)\right], \end{array}$$

where *i* = 1, 2, ⋯, *N* − (*m* − 1)*τ*, *x* is the signal with *N* samples, and *X* is the *m*-dimensional vector. Afterwards, the correlation integral of *X* is defined as the probability that two points of the set are in the same partition of size *r*. It is obtained using the following equation:

(13) $$\begin{array}{c} C\left(r\right)=\frac{2}{N\left(N-1\right)}\underset{i\neq j}{\sum }\phi \left(r-\left|X\left(i\right)-X\left(j\right)\right|\right), \end{array}$$

where *C*(*r*) and *ϕ* represent the correlation integral and the Heaviside step function, respectively. In the next phase, (14) is utilized to obtain the raw correlation dimension.

(14) $$\begin{array}{c} D=\underset{r⟶0}{\lim}\frac{\ln C\left(r\right)}{\ln\left(r\right)}. \end{array}$$

Finally, the different values of *D* are computed using (14) for the incremental value of *m*. This process causes a gradual of *D*, and eventually, *D* reaches saturation. The saturated value of *D* is considered as the estimated correlation dimension of the signal

(d) *Lyapunov exponent*: the chaos of a dynamic system is quantified by the Lyapunov exponent, which estimates the development or decay rate of minor perturbations along each major axis of the phase space system [38]. Consider a dynamic system with the *d* dimension. It is possible to determine the *d* number of Lyapunov exponents for this system. However, in the majority of real-world applications, the greatest Lyapunov exponent (LLE) is regarded as the extracted feature by the Lyapunov exponent. A dynamic system's maximal Lyapunov exponent (*λ*_1_) is defined as follows:

(15) $$\begin{array}{c} d_{j}\left(i\right)=d_{j}\left(0\right)\exp\left(\lambda_{1}i\Delta t\right), \end{array}$$

where *d*_*j*_(*i*) denotes the mean Euclidian distance between two neighbor trajectories at *i* time and *d*_*j*_(0) represents the Euclidian distance between the *j*th pair of initially most adjacent neighbors after *i* time. In order to compute the LLE, the following equation is used:

(16) $$\begin{array}{c} y\left(i\right)=\frac{1}{\Delta t}<\ln\left(d_{j}\left(i\right)\right)>, \end{array}$$

where *y*(*i*) and <ln(*d*_*j*_(*i*))> represents the approximated LLE and the average value of the natural logarithm of *d*_*j*_(*i*) over all values of *j*, espectively

(e) *C0-complexity*: it is a measure that is aimed at quantifying irregularities of a signal by defining the ratio of the irregular components to the original signal [39]. Consider a signal *x*(*n*) with the *N* number of samples. Firstly, the fast Fourier transform of the *x*(*n*) (*X*(*k*)) is computed and the average value of the magnitude of *X*(*k*) (*M*) is obtained as follows:

(17) $$\begin{array}{c} M=\frac{1}{N}\overset{N-1}{\underset{k=0}{\sum }}{\left|X\left(k\right)\right|}^{2}. \end{array}$$

Now, a spectrum called *Y*(*k*) is constructed using *X*(*k*) and *M* as follows:

(18) $$\begin{array}{c} Y\left(k\right)=\left\{\begin{array}{cc} X\left(k\right), & {\left|X\left(k\right)\right|}^{2}>M,\\ 0, & {\left|X\left(k\right)\right|}^{2}<M. \end{array}\right. \end{array}$$

By applying inverse Fourier transform to *Y*(*k*), *y*(*n*) is obtained and the C0-complexity of the *x*(*n*) is provided as follows:

(19) $$\begin{array}{c} C0=\frac{A_{1}}{A_{0}}=\frac{\sum_{n=0}^{N-1}{\left|x\left(n\right)-y\left(n\right)\right|}^{2}}{\sum_{n=0}^{N-1}{\left|x\left(n\right)\right|}^{2}}, \end{array}$$

where *C*0, *A*_1_, and *A*_0_ represent C0-complexity, the power of irregular, and regular parts of *x*(*n*),respectively

(f) *Kolmogorov entropy*: it reflects the loss of information's rate of a signal to quantify its chaotic degree [40]. In order to compute it, an equation based on the average rate of the loss of information of a signal with *n* samples is defined as follows:

(20) $$\begin{array}{c} \text{KE}=-\underset{\tau ⟶0}{\lim}\underset{\varepsilon ⟶0}{\lim}\underset{n⟶\infty }{\lim}\frac{1}{n\tau }\underset{i_{0}\cdots i_{n-1}}{\sum }P_{i_{0}\cdots i_{n-1}}\ln\left(P_{i_{0}\cdots i_{n-1}}\right), \end{array}$$

where *P*_*i*_0_⋯*i*_*n*−1__ and KE denote the loss of information per each sample and estimated Kolmogorov entropy, respectively. It is worth mentioning that the positive and finite value of KE represents that the dynamic phenomena in the signal are chaotic. Moreover, the zero value indicates that the signal contains regular phenomena and infinite KE corresponds with the existence of nondeterministic phenomena in the signal

(g) *Shannon entropy*: it is another metric for quantifying the chaotic rate of a signal, proposed by Shannon [41]. Given a signal with *N* samples, the Shannon entropy is defined as follows:

(21) $$\begin{array}{c} H=-\overset{N}{\underset{i=1}{\sum }}p_{i}\ln\left(p_{i}\right), \end{array}$$

where *H* and *p*_*i*_ represent the Shannon entropy of the signal and the probability of having the *i* sample in the signal, respectively

(h) *Approximate entropy*: it is an algorithm to estimate the rate of regularity and the unpredictability of fluctuations of a signal [42]. If this estimation is higher, the signal contains more irregularity. In the first step of this algorithm, a sequence of vectors (*X*(*i*)) is constructed from a signal as follows:

(22) $$\begin{array}{c} X\left(i\right)=\left[x\left(i\right),x\left(i+1\right),\cdots ,x\left(i+m-1\right)\right],1\leq i\leq N-m+1, \end{array}$$

where *x*(*n*) is the signal with *N* samples. In the next phase, the distance between *X*(*i*) and *X*(*j*) (*D*[*X*(*i*)), *X*(*j*)]) is computed using the following equation:

(23) $$\begin{array}{c} D\left[X\left(i\right),X\left(j\right)\right]=\underset{k=1,2,\cdots ,m}{\max}\left[\left|x\left(i+k-1\right)-x\left(j+k-1\right)\right|\right], \end{array}$$

where |.| is the Euclidean distance. Now, *C*_*i*_^*m*^(*r*) is calculated for each *i*, *i* = 1, 2, ⋯, *N* − *m* as follows:

(24) $$\begin{array}{c} C_{i}^{m}\left(r\right)=\frac{\text{number of }D\left[X\left(i\right),X\left(j\right)\right]\leq r}{N-m-1}, \end{array}$$

where *r* denotes the threshold for *D*[*X*(*i*), *X*(*j*)]. Finally, the approximate entropy (ApEn) is determined as follows:

(25) $$\begin{array}{c} \text{ApEn}=\Phi^{m}\left(r\right)-\Phi^{m+1}\left(r\right), \end{array}$$

where *Φ*^*m*^(*r*) is defined as follows:

(26) $$\begin{array}{c} \Phi^{m}\left(r\right)=\frac{1}{N-m-1}\overset{N-m-1}{\underset{i=1}{\sum }}\ln\left(C_{i}^{m}\left(r\right)\right) \end{array}$$

In this work, the values of *m* and *r* were set to 2 and 0.2var(*x*), respectively.

The article "Automatic Diagnosis of Mild Cognitive Impairment Based on Spectral, Functional Connectivity, and Nonlinear EEG-Based Features" was published in 2022. Journal: Comput Math Methods Med.

The amount of features in each feature set in the suggested methods is displayed in Table 1. Table 1 shows that the spectral, functional connectivity, and nonlinear feature sets, comprising 108, 171, and 152 characteristics, respectively. It is important to note that the aforementioned features are vectorially concatenated to provide a vector for each data. There are 19 features in each frequency subband power. We recovered 8 features for theta, alpha, beta, and theta frequency subbands for the IA feature. 32 features were therefore included in the IA. Additionally, each nonlinear feature has 19 features.

#### 2.2.3. Feature Selection

In machine learning frameworks, the goal of feature selection is to find the best subset of features to improve the classification performance by ignoring irrelevant and redundant attributes. In this study, a wrapper feature selection algorithm called SBFS was employed to obtain the best features' subset for discriminating MCI and HC samples. The main steps of the SBFS algorithm are illustrated in Algorithm 1. Briefly, SBFS attempts to obtain the best features' subset by sequentially eliminating features from the entire feature set. As shown in Algorithm 1, removing features continues as long as the objective criterion is ascending [43]. In this work, the criterion (*J*) is set to the average accuracy in 10-fold crossvalidation. It should be mentioned that the classifier of the SBFS method was set to linear discriminant analysis (LDA) in our study.

#### 2.2.4. Classification

The main component of supervised machine learning frameworks is classification, which is aimed at predicting a class label or a specific example of incoming data. Classification models carry out this task. The classification model for the suggested machine learning framework was chosen by comparing a number of them in this study, including SVM with linear (LSVM) and radial basis function (RBFSVM) kernels, LR, KNN, decision tree (DT), naive Bayes (NB), RUSBoost (RB), and GentleBoost (GB). Additionally, before training and testing classifiers, the training and testing sets were applied to the *z*-score transformation. Finding the optimum decision boundary that can categorize an n-dimensional feature space into classes is the primary objective of SVM models. A hyperplane and a hyper radial basis curve are the ideal decision boundaries for LSVM and RBFSVM, respectively. The extreme points or vectors selected by these models aid in determining the optimal decision boundary. Support vectors are used to describe these severe situations. A nonparametric supervised learning technique that makes advantage of neighbor similarity is the KNN algorithm. A class membership is the result of this method. A datum is assigned to the class that has the highest percentage of support from its *k* closest neighbors after receiving a majority vote from those neighbors. A DT method is a decision-support tool that categorizes each item class using a tree-like model of decisions and their potential outcomes. A subset of probabilistic classifiers called NB is based on the Bayes theorem and assumes independence between sample features. On ensemble classifiers, the RB and GB models are built. Using different base models as a starting point, ensemble learning creates a new classifier that outperforms all of its component classifiers. The Bayesian optimizer was also utilized to optimize the hyperparameters of LSVM, RBFSVM, LR, DT, NB, RB, and GB models.

The article "Automatic Diagnosis of Mild Cognitive Impairment Based on Spectral, Functional Connectivity, and Nonlinear EEG-Based Features" was published in 2022. Journal: Comput Math Methods Med.

#### 2.2.5. Validation

The 10-fold crossvalidation strategy was utilized in this work to assess the classification performance of the suggested MCI diagnosis method. This method divides the dataset into 10 folds at random. The model is then trained using a subset of 9 folds as the training set and validated using a subset of 1 fold as the testing set. To make each fold the testing subset once, this procedure is repeated ten times. The classification performance of the suggested method may be assessed using the accuracy (AC), sensitivity (SE), specificity (SP), F1-score (F1), and false discovery rate (FDR) performance metrics by applying the testing set to the trained model and comparing the predicted and actual labels. The following is how the aforementioned metrics are calculated:

(27) $$\begin{array}{c} \text{AC}=\frac{\text{TP}+\text{TN}}{\text{TP}+\text{FN}+\text{TN}+\text{FP}},\\ \text{SE}=\frac{\text{TP}}{\text{TP}+\text{FN}},\\ \text{SP}=\frac{\text{TN}}{\text{FP}+\text{TN}},\\ \text{F}1=\frac{2\text{TP}}{2\text{TP}+\text{FP}+\text{FN}},\\ \text{FDR}=\frac{\text{FP}}{\text{FP}+\text{TN}}, \end{array}$$

where TP is the number of MCI cases that are correctly predicted, FN is the number of MCI cases that are incorrectly predicted as HC samples, FP is the number of HC cases that are incorrectly predicted as MCI cases, and TN is the number of HC samples that are correctly predicted.

## 3. Results

This section evaluates the performance of the suggested framework from a number of angles. The obtained results of the classification models using the suggested strategy are provided in the first portion in order to choose the best of them. The next step was to select the ideal combination for the suggested framework by using each set of attributes and their combinations as the input framework. Then, in order to examine the difference between the two groups based on the aforementioned features, the EEG signal strength disparities in the alpha, beta, theta, and delta frequency subbands as well as the most important functional connectivity features between MCI and HC cases are investigated. The EEG signal band powers and functional connectivity feature sets, among the recovered feature sets in this study, may offer some biological notions of MCI. To ascertain which EEG signal band powers and functional connectivity coefficients most significantly differ between MCI and HC subjects, we presented these sections. The intersection of the returned subsets by SBFS in the execution of the suggested framework's 10-fold crossvalidation is then reported and examined. Finally, a report and analysis of the leave-one-participant-out crossvalidation approach's acquired results for the suggested framework was made.

The article "Automatic Diagnosis of Mild Cognitive Impairment Based on Spectral, Functional Connectivity, and Nonlinear EEG-Based Features" was published in 2022. Journal: Comput Math Methods Med.

### 3.1. Results per Classifiers

The outcomes of the proposed framework employing the aforementioned classification models are listed in Table 2. According to Table 2's findings, LSVM had the best classification performance. The given framework utilized the LSVM model to achieve an average AC of 99.4%, SE of 98.8%, SP of 100%, F1 of 99.4%, and FDR of 0%. Comparing this classifier to the others, it produced results with higher means for AC, SP, and F1 and a lower mean for FDR. Additionally, it outperformed the other classification models in terms of performance measures with the lowest standard deviation, demonstrating the greater stability of its performance within the framework that was presented. According to the results in Table 2, KNN and RBFSVM were the second and third best classification models in the framework that was provided. In comparison to other classifiers, RBFSVM earned the SP metric's greatest mean and lowest standard deviation. With the lowest mean of AC, SE, and F1 metrics among the employed classifiers, NB offered the worst classification performance. The classification performance of the other classifiers, including RB, GB, DT, and LT, was comparable. The box plots of the AC, SE, SP, and F1 metric-achieved values by the proposed framework utilizing classification models are shown in Figure 2. As depicted in Figure 2, the acquired AC, SE, SP, and F1 metric values of LSVM, KNN, and RBFSVM were reasonably high, confirming that the suggested method's use of these classifiers produced acceptable performance. LSVM outperformed the other classifiers in terms of AC, SE, SP, and F1 performance metrics. Additionally, LSVM's boxplots for the aforementioned metrics were less negative than those for other classifiers. These findings show that, in terms of classification accuracy and performance resilience, the LSVM model is better to alternative classifiers for the suggested framework. Overall, the findings showed that LSVM, KNN, and RBFSVM were the three best classifiers for the suggested framework. The receiver operator characteristic (ROC) curves for each classification model in the proposed framework are shown in Figure 3. DT, GB, KNN, LSVM, LR, NB, RB, and RBFSVM had areas under the curve (AUC) of 0.85, 0.86, 0.98, 0.99, 0.92, 0.87, 0.65, and 0.99, respectively. These findings showed that employing the LSVM and RBFSVM classification models, the proposed framework had the best classification performance.

The article "Automatic Diagnosis of Mild Cognitive Impairment Based on Spectral, Functional Connectivity, and Nonlinear EEG-Based Features" was published in 2022. Journal: Comput Math Methods Med.

### 3.2. Results per Feature Set

The optimal input for the suggested framework was chosen in this part using each feature set and its combinations as the input classification framework. It is important to note that the three top classifiers from the previous section carried out these evaluations. The classification outcomes of the proposed framework employing each input and the LSVM, RBFSVM, and KNN classification models are shown in Table 3. Based on the reported results in Table 3, the integration of functional connectivity, spectral, and nonlinear feature sets provided the best classification performances by obtaining the highest average of AC, SE, SP, and F1 parameters and the lowest means of the FDR metric. Additionally, as compared to the other inputs, the integration of the aforementioned feature sets yielded the lowest standard deviations of evaluation metrics, proving that the proposed framework is more reliable when all EEG feature sets are used as input. LSVM, which delivered an average AC of 99.4%, SE of 98.8%, SP of 100%, F1 of 99.4%, and FDR of 0%, provided the best classification performance of the suggested framework employing the combination of functional connectivity, spectral, and nonlinear feature sets. Performance was nearly identical when functional connectivity was combined with the spectral and nonlinear feature sets. In terms of classification accuracy performance, these combinations come in second. KNN achieved an average AC of 98.8%, SE of 98.7%, SP of 97.5%, F1 of 98.9%, and FDR of 0.6%, which was the best classification performance of the suggested framework employing the combination of functional connectivity and spectral feature sets. KNN also offered the best classification performance for the combination of functional connectivity and nonlinear feature sets, with an average AC of 98.8%, SE of 100.0%, SP of 97.0%, F1 of 99.0%, and FDR of 1.8%. In terms of performance for classification accuracy, these combinations come in second. The suggested framework's functional connectivity and spectral feature set combination produced the best classification results when utilizing KNN, which had an average AC of 98.8%, SE of 98.7%, SP of 97.5%, F1 of 98.9%, and FDR of 0.6%. With an average AC of 98.8%, SE of 100.0%, SP of 97.0%, F1 of 99.0%, and FDR of 1.8%, KNN also offered the greatest classification performance for the combination of functional connectivity and nonlinear feature sets. These pairings are in second place for categorization accuracy performance. KNN achieved the best classification results of the suggested framework employing the combination of functional connectivity and spectral feature sets, with an average AC of 98.8%, SE of 98.7%, SP of 97.5%, F1 of 98.9%, and FDR of 0.6%. KNN also offered the best classification performance for the combination of functional connectivity and nonlinear feature sets, with an average AC of 98.8%, SE of 100.0%, SP of 97.0%, F1 of 99.0%, and FDR of 1.8%.

The article "Automatic Diagnosis of Mild Cognitive Impairment Based on Spectral, Functional Connectivity, and Nonlinear EEG-Based Features" was published in 2022. Journal: Comput Math Methods Med.

### 3.3. EEG Signal Power Analysis

This section looked into the changes in alpha, theta, beta, and delta EEG band power between MCI and HC samples at various scalp locations. In order to quantify the difference between the two groups by these band powers, the band powers of the aforementioned frequency subbands for MCI and HC cases were studied using the *t*-test approach.  Table 4 provides the *t*-test results on the alpha, theta, beta, and delta EEG signal powers of MCI and HC cases in each EEG channel. According to these results, alpha and beta band powers provided the most significant difference between MCI and HC cases. Using alpha and beta band powers, the frontal, parietal, and temporal regions of the scalp offered greater discrimination than other regions. Theta power was the next-best EEG band power for MCI and HC discriminating. However, the delta band power was unable to distinguish significantly between the MCI and HC patients.  Figure 4 displays the alpha, delta, beta, and theta band powers on the EEG topographic maps of HC and MCI subjects. According to Figure 4, the frontal lobe used alpha band power to significantly distinguish between HC and MCI individuals. The frontal, temporal, and occipital lobes contributed significantly to the variations between HC and MCI subjects in theta band power. The major differences between HC and MCI subjects employing beta band power were found in the left temporal and occipital areas. The frontal and occipital areas supplied the substantial variations between HC and MCI subjects for delta band power.

### 3.4. Functional Connectivity Analysis

The major objective of this section is to use the *t*-test approach to identify the most important functional connectivity coefficients that distinguish between HC and MCI cases. In order to achieve this, the *p* value metric of the *t*-test method was used to rank the functional connectivity coefficients of MCI and HC cases and the top 10 values were identified. The top ten functional coefficients for distinguishing between HC and MCI samples are listed in Table 5 along with associated *p* value metrics. These findings show that there is a significant difference between the classes utilizing each of the top ten functional connectivity measures, with the statistical significance difference of the ten features between MCI and HC cases being less than 1*e* − 3. The F3-C3, Fp1-F3, F3-T5, P3-F7, P4-Cz, C3-O1, C3-C4, Fp1-Fp2, C3-Fp2, and Fz-C4 were the top 10 features which provided the most significant difference between HC and MCI classes among functional connectivity coefficients. The boxplot of the top ten functional connectivity features for MCI and HC cases is shown in Figure 5. These boxplots show that there can be large disparities between MCI and HC samples depending on these top ten features. The functional connection between the frontal, temporal, central, and parietal scalp regions is also inferred from these findings to have contributed to the most notable disparities between MCI and HC classes.

The article "Automatic Diagnosis of Mild Cognitive Impairment Based on Spectral, Functional Connectivity, and Nonlinear EEG-Based Features" was published in 2022. Journal: Comput Math Methods Med.

### 3.5. Selected Features

In the evaluation of the proposed framework using 10-fold crossvalidation, the SBFS method returns a specific subset of features as selected features in each iteration, which resulted in 10 subsets of features for all iterations. The intersection of these ten subsets is reported and examined in this subsection. The details of these traits are listed in Table 6. These features totaled 361 and were divided into three sets: the spectral set (108), the functional connectivity set (171), and the nonlinear set (82). These results show that all spectral and functional connectivity features were chosen in all iterations of 10-fold crossvalidation and had the biggest proportion of the features chosen, whereas 82 nonlinear characteristics were chosen in all iterations.

### 3.6. Participant-Independent Evaluation

The suggested framework was validated using the leave-one-participant-out crossvalidation approach in order to be assessed from the standpoint of the participant independence. In this method, the spectral, nonlinear, and functional connectivity properties were retrieved from each participant's EEG signals without segmenting them first. The remaining data were then utilized as the training set, with one data set serving as the testing set. Until each case was used as the testing set, this was reproduced 34 times. The classification model for the proposed framework in this evaluation was an LSVM classifier. The resulting confusion matrix by the suggested framework in this assessment is shown in Table 7. Table 7 shows that the suggested framework used an LSVM model to achieve an AC of 91.1%, SE of 88.8%, SP of 93.7%, F1 of 91.4%, and FDR of 5.8%. These findings show that even in more demanding evaluations like the leave-one-participant-out cross-validation strategy, the suggested framework provided an accurate and acceptable classification performance.

The article "Automatic Diagnosis of Mild Cognitive Impairment Based on Spectral, Functional Connectivity, and Nonlinear EEG-Based Features" was published in 2022. Journal: Comput Math Methods Med.

## 4. Discussion

This paper presents a machine learning framework for MCI diagnosis based on EEG signals using spectral, functional connectivity, and nonlinear features. The findings demonstrate how well the proposed framework performs accurate and reliable classification. The spectral and functional connectivity feature sets outperformed the nonlinear feature set among the feature sets. This may be due to the fact that nonlinear feature sets are less likely than spectral and functional connectivity feature sets to distinguish between MCI and HC patients. These feature sets may also offer biological explanations for cognitive states. This study used the *t*-test method to examine the band powers of the alpha, delta, beta, and theta frequency subbands in each EEG channel of MCI and HC individuals. This test revealed that the most important distinction between MCI and HC cases was between alpha and beta band powers. Beta band power is more connected to the traits of MCI and other types of dementia than alpha band power. The relationship between beta band power and several MCI-related cognitive processes, including as expectation, consciousness, memory, and problem-solving, may account for the physiological differentiation made by beta band power. Furthermore, the differentiation made by alpha band power may be linked to further MCI-related cognitive states, such as difficulty focusing and extreme relaxation. Additionally, the top 10 functional connectivity characteristics distinguished between the HC and MCI groups in statistical analysis of the MCI and HC samples were presented. The findings show that the most effective way to distinguish between MCI and HC cases is through the functional connectivity coefficients across the frontal, temporal, central, and parietal scalp areas. These findings may be the result of a correlation between certain MCI-related mental states and cognitive tasks, such as elicitation, attention, thinking, problem-solving, and memory-related processes and the linkages between frontal, temporal, central, and parietal regions.

A comparison of the proposed framework and earlier studies for MCI diagnosis based on EEG data is shown in Table 8. It should be noted that only [19, 21] research utilized the same dataset and evaluation process for their approaches but the content and methodologies of other publications are not the same as our work. The given framework, which has the highest mean of AC among state-of-the-art methods, outperforms the other state-of-the-art strategies for automatic MCI diagnosis based on EEG signals, according to the results described in Table 8. The fundamental improvement of the proposed framework over earlier research is the integration of the spectral, functional connectivity, and nonlinear properties, which have not been combined in such a way in other works. According to the results, the combination of spectral, functional connectivity, and nonlinear features produced the greatest classification results, exceeding earlier studies that predicated MCI diagnosis on EEG data. Another significant distinction between the proposed framework and earlier research is that the provided framework uses the SBFS algorithm as a feature selection strategy, whereas earlier works employed other feature selection approaches including RF and rank-based feature selection methods.

The article "Automatic Diagnosis of Mild Cognitive Impairment Based on Spectral, Functional Connectivity, and Nonlinear EEG-Based Features" was published in 2022. Journal: Comput Math Methods Med.

The main restriction is the tiny sample size of the used dataset. As a result, the proposed method's precise and reliable performance could not be highly generalizable. By dividing each EEG signal into five-minute chunks, we did our best to make up for this restriction. However, further MCI EEG datasets are necessary for the applicability of this paradigm and related strategies. On the other hand, there are very few publicly available MCI EEG datasets with more participants. It is advantageous to generalize the validation of the suggested methodologies because public datasets generally have the potential to open up new avenues for collaboration. The framework that is being given also has a heavy computational load. The method's computing load was raised even though the integration of all feature sets produced the maximum classification accuracy and produced a high-dimensional feature matrix. It further complicates how the framework should be interpreted in terms of physiological and biomarker characteristics. Additionally, it is unclear how clinically applicable this study and all automatic EEG-based MCI detection methods are. More clinical experimental evidence is required to confirm these techniques' clinical efficacy.

However, this paper proposes an automated MCI diagnosis framework based on EEG signals with an accurate and robust classification performance according to the obtained results. It could be developed to use it as a computer-aided diagnosis (CAD) tool for clinical purposes. Future studies can also focus on providing more MCI EEG datasets and implementing deep learning approaches for automatic EEG-based MCI diagnosis.

The article "Automatic Diagnosis of Mild Cognitive Impairment Based on Spectral, Functional Connectivity, and Nonlinear EEG-Based Features" was published in 2022. Journal: Comput Math Methods Med.

## 5. Conclusion

This study provided a spectral, functional connectivity, and nonlinear feature-based machine learning framework for automatic MCI diagnosis. In this framework, SBFS was applied as a feature selection approach to choose the best subset of features and enhance classification performance. Additionally, many categorization models were assessed in order to choose the best one for the suggested framework. The optimal input for the proposed MCI diagnosis framework was also determined by applying each of the feature sets and their combinations to the proposed framework. Based on the obtained results, the LSVM classifier combined with functional connectivity, spectral, and nonlinear feature sets achieved the best classification performance of the proposed framework, which provided an average AC of 99.4%, SE of 98.8%, SP of 100%, F1 of 99.4%, and FDR of 0%. Additionally, the leave-one-participant-out crossvalidation method was used to evaluate the offered framework. The results showed that the LSVM model had an AC of 91.1%, SE of 88.8%, SP of 93.7%, F1 of 91.4%, and FDR of 5.8%. These findings demonstrate how well the newly presented framework performs accurate and reliable classification. The current methodology offered a superior classification performance in terms of robustness and accuracy when compared to earlier research for EEG-based automatic MCI diagnosis. Based on the results, the medical equipment businesses would be encouraged to create a CAD system for MCI diagnosis utilizing the same proposed framework due to the high potential of the given framework to identify MCI patients. Future research can concentrate on supplying additional MCI EEG datasets and utilizing cutting-edge deep learning techniques for automatic EEG-based MCI diagnosis.

## Figures and Tables

**Figure 1:** Overview of the proposed EEG-based methodology for MCI diagnosis.

**Figure 2:** The box plots of the obtained values of AC (a), SE (b), SP (c), and F1 (d) metrics per classifier using the 10-fold crossvalidation method.

**Figure 3:** The ROC plots of the proposed framework per classifier using the 10-fold crossvalidation method.

**Figure 4:** The EEG topographic maps of HC and MCI cases in terms of the alpha, delta, beta, and theta band powers.

**Figure 5:** The boxplot of ten top functional connectivity features of MCI and HC cases.

**Algorithm 1:** The SBFS algorithm.

**Table 1:** The more details of each feature set.

Feature set	Number of features
Functional connectivity	108
Spectral	171
Nonlinear	152

**Table 2:** The obtained results of the proposed framework using different classifiers in terms of the percentage (%) of the mean and standard deviation of AC, SE, SP, F1, and FDR metrics.

Classifier	AC (mean ± Std)	SE (mean ± Std)	SP (mean ± Std)	F1 (mean ± Std)	FDR (mean ± Std)
LSVM	99.4 ± 1.8	98.8 ± 3.5	100 ± 0	99.4 ± 1.8	0 ± 0
RBFSVM	95.9 ± 3.9	100 ± 0	91.1 ± 8.4	96.3 ± 3.6	6.8 ± 6.7
LR	87.8 ± 4.2	85.2 ± 11.6	90.0 ± 10.8	87.5 ± 5.5	8.2 ± 8.7
KNN	98.2 ± 2.8	97.5 ± 5.6	98.7 ± 3.9	98.1 ± 3.2	1.0 ± 3.1
DT	80.2 ± 8.8	79.3 ± 15.6	81.6 ± 15.2	80.1 ± 10.1	16.8 ± 11.7
GB	81.4 ± 7.1	81.0 ± 13.1	81.8 ± 10.5	81.2 ± 9.4	17.3 ± 9.8
NB	77.4 ± 7.3	63.2 ± 15.2	92.5 ± 7.0	73.4 ± 11.9	9.9 ± 9.6
RB	86.6 ± 10.3	85.8 ± 9.4	87.0 ± 16.5	87.3 ± 87.3	10.5 ± 11.1

The article "Automatic Diagnosis of Mild Cognitive Impairment Based on Spectral, Functional Connectivity, and Nonlinear EEG-Based Features" was published in 2022. Journal: Comput Math Methods Med.

**Table 3:** The classification results of the proposed method based on RBFSVM, LSVM, and KNN classification models using different EEG feature sets in terms of the percentage (%) of the mean and standard deviation of AC, SE, SP, F1, and FDR metrics.

Feature set	Classifier	AC (mean ± Std)	SE (mean ± Std)	SP (mean ± Std)	F1 (mean ± Std)	FDR (mean ± Std)
Functional connectivity + spectral + nonlinear	LSVM	99.4 ± 1.8	98.8 ± 3.5	100.0 ± 0.0	99.4 ± 1.8	0.0 ± 0.0
	RBFSVM	95.9 ± 3.9	100.0 ± 0.0	91.1 ± 8.4	96.3 ± 3.6	6.8 ± 6.7
	KNN	98.2 ± 2.8	97.5 ± 5.6	98.7 ± 3.9	98.1 ± 3.2	1.0 ± 3.1
Functional connectivity + nonlinear	LSVM	98.8 ± 2.4	98.7 ± 3.9	99.0 ± 3.1	98.7 ± 2.6	1.1 ± 3.5
	RBFSVM	94.8 ± 5.6	100.0 ± 0.0	89.3 ± 10.8	95.2 ± 5.3	8.6 ± 9.3
	KNN	98.8 ± 2.4	100.0 ± 0.0	97.0 ± 6.7	99.0 ± 2.1	1.8 ± 4.0
Functional connectivity + spectral	LSVM	98.8 ± 2.4	98.5 ± 4.5	98.8 ± 3.5	98.6 ± 2.8	1.1 ± 3.5
	RBFSVM	97.1 ± 4.1	100.0 ± 0.0	93.2 ± 9.8	97.2 ± 3.9	6.5 ± 7.9
	KNN	98.8 ± 2.4	98.7 ± 3.9	97.5 ± 7.9	98.9 ± 2.2	0.6 ± 2.1
Spectral + nonlinear	LSVM	94.1 ± 5.5	95.9 ± 6.8	91.8 ± 9.9	94.6 ± 4.7	6.0 ± 7.1
	RBFSVM	94.2 ± 7.2	99.0 ± 2.8	88.7 ± 17.6	94.6 ± 6.1	8.6 ± 11.0
	KNN	98.2 ± 3.9	98.0 ± 4.2	98.5 ± 4.5	98.4 ± 3.4	1.0 ± 3.1
Spectral	LSVM	93.0 ± 7.9	92.3 ± 9.5	93.8 ± 8.1	93.2 ± 8.5	5.6 ± 8.4
	RBFSVM	95.3 ± 3.6	99.0 ± 3.1	90.6 ± 9.1	95.8 ± 3.2	6.7 ± 6.4
	KNN	98.8 ± 2.4	98.0 ± 4.2	100.0 ± 0.0	98.9 ± 2.2	0.0 ± 0.0
Functional connectivity	LSVM	97.6 ± 4.9	100.0 ± 0.0	95.1 ± 10.4	97.8 ± 4.6	3.8 ± 8.3
	RBFSVM	98.1 ± 2.5	97.7 ± 3.4	98.6 ± 2.3	98.2 ± 2.3	1.2 ± 2.1
	KNN	97.0 ± 2.6	96.8 ± 3.7	96.1 ± 3.8	96.7 ± 2.4	3.2 ± 2.9
Nonlinear	LSVM	86.7 ± 8.6	86.9 ± 9.4	86.5 ± 13.6	86.5 ± 9.5	12.9 ± 13.6
	RBFSVM	83.8 ± 11.3	89.1 ± 12.9	78.7 ± 16.4	84.2 ± 12.6	19.1 ± 15.1
	KNN	87.4 ± 8.1	85.2 ± 11.8	91.7 ± 11.4	87.1 ± 9.2	8.9 ± 12.5

**Table 4:** The *t*-test results on the alpha, theta, beta, and delta EEG band powers in each EEG channel. Italic items indicate *p* value <0.01.

Brain region	EEG channel	Alpha *p* value	Beta *p* value	Delta *p* value	Theta *p* value
Frontal	Fp1	0.9474	0.2499	0.3600	0.9732
	Fp2	0.1083	0.0267	0.5997	0.3103
	F7	0.2214	0.3346	0.2985	0.2593
	F3	0.0871	0.1177	0.2291	0.2874
	Fz	*0.0001*	*0.0001*	0.0863	*0.0032*
	F4	*0.0011*	*0.0091*	0.3181	0.0335
	F8	*0.0001*	*0.0001*	0.0241	*0.0005*
Central	C3	0.2783	0.6267	0.4596	0.2667
	Cz	*0.0069*	*0.0001*	0.0527	0.0174
	C4	0.2179	0.0588	0.8330	0.5390
Occipital	O1	0.0301	0.0300	0.1801	0.1105
	O2	*0.0001*	*0.0001*	*0.0031*	*0.0001*
Parietal	P3	0.1187	0.7611	0.5157	0.3680
	P4	*0.0036*	*0.0001*	*0.0049*	*0.0014*
	Pz	*0.0051*	*0.0001*	*0.1577*	*0.0078*
Temporal	T3	0.6706	0.4975	0.4047	0.4661
	T5	0.0231	*0.0060*	0.1148	0.0863
	T4	*0.0033*	*0.0061*	0.0409	0.0164
	T6	*0.0006*	*0.0002*	0.0772	*0.0068*

The article "Automatic Diagnosis of Mild Cognitive Impairment Based on Spectral, Functional Connectivity, and Nonlinear EEG-Based Features" was published in 2022. Journal: Comput Math Methods Med.

**Table 5:** Ten top functional connectivity features in terms of discrimination between HC and MCI classes with their *p* values of the *t*-test method.

Functional connectivity feature	*t*-test *p* value
F3-C3	6.46*e* − 08
Fp1-F3	1.12*e* − 06
F3-T5	3.97*e* − 06
P3-F7	2.63*e* − 05
P4-Cz	5.09*e* − 05
C3-O1	1.18*e* − 04
C3-C4	1.22*e* − 04
Fp1-Fp2	1.75*e* − 04
C3-Fp2	2.34*e* − 04
Fz-C4	3.47*e* − 04

**Table 6:** The intersection of the selected features in all iterations of 10-fold crossvalidation.

Feature set	Selected features
Functional connectivity	All features
Spectral	All features
Nonlinear	DFA (Fp1, Fp2, F4, Fz, T4, T6, Pz, O1, O2)
	Higuchi (Fp2, F8, T4, P4, Pz, O2, C4, Cz, O2)
	Correlation dimension (Fp1, Fp2, F3, Fz, T3, T4, T6, P3, C3, C4, O1, O2)
	Lyapunov exponent (F3, F4, Fz, T5, P4, O2, C3, C4, Cz, O1, O2)
	C0-complexity (Fp1, F4, T3, P3, P4, Pz, C4, O1)
	Kolmogorov entropy (Fp1, Fp2, F3, F8, T3, T5, T6, Pz, C4, O1, O2)
	Shannon entropy (Fp1, Fp2, F3, Fz, T3, T6, T4, T5, O1, Cz)
	Approximate entropy (Fp1, Fp2, F4, F3, Fz, F7, T6, P3, P4, O2, C3, Cz)

**Table 7:** The obtained confusion matrix by the proposed framework using the leave-one-participant-out cross-validation approach.

		True classes	
		MCI	HC
Predicted classes	MCI	16	1
	HC	2	15

**Table 8:** Comparison between the proposed framework and previous works for identifying MCI patients based on EEG signals.

Study	Year	EEG features	Classifiers	Reported AC
[19]	2016	Spectral features	NF and KNN	88.8%
[21]	2019	Time series signal spectral and features	LC-KSVD and CLC-KSVD	88.9%
[22]	2019	Time and spectral domain features	LR and SVM	87.9%
[23]	2019	Spectral-temporal features	SVM	96.94%
[24]	2019	Spectral, statistical, and nonlinear features	SVM	96.94%
[26]	2020	AR and PE features	ELM, SVM, and KNN	97.64%
Proposed framework	2021	Spectral, functional connectivity and,	LINSVM, RBFSVM, and LR,	99.4%
		Nonlinear features	DT, RB, NB, GB, and KNN	

The article "Automatic Diagnosis of Mild Cognitive Impairment Based on Spectral, Functional Connectivity, and Nonlinear EEG-Based Features" was published in 2022. Journal: Comput Math Methods Med.

## Data Availability

The used dataset in this study is a public dataset. The data statement was cheked and it is valid.
